# Research on Data Analysis Network of TCM Tongue Diagnosis Based on Deep Learning Technology

**DOI:** 10.1155/2022/9372807

**Published:** 2022-03-29

**Authors:** Zongrun Li, Xiujuan Ren, Lin Xiao, Jing Qi, Tianli Fu, Weihong Li

**Affiliations:** ^1^Basic Medical College, Chengdu University of TCM, Chengdu, China; ^2^School of Rehabilitation Medicine, Weifang Medical University, Weifang, China; ^3^Administrative Office of Weifang People's Hospital, Weifang, China; ^4^Basic Medical College, Weifang Medical University, Weifang, China; ^5^School of Management, Weifang Medical University, Weifang, China

## Abstract

The aim of the study is to build a tongue image intelligent analysis “end-to-end” deep learning network based on a tongue diagnosis image of traditional Chinese medicine. The tongue target region in the original image was segmented by the UNet tongue segmentation model at the front end of the network. After segmentation, the feature vector of the tongue target region was extracted by the ResNet network, and then the blood pressure on the day of shooting was fused with the feature vector extracted by the ResNet network through the convolution operation method to complete the extraction of two groups of data of tongue feature and fusion feature. Based on analyzing the data of blood pressure, tongue image, and their fusion at the end of the network, four regression analysis methods were used to predict the stage mean value. After training, the model is tested with the test set data, and the test results are evaluated with mean absolute error (MAE). The prediction error of the model based on the fusion data of tongue image and blood pressure on the day of shooting was lower than that of the other two data modes. The UNet tongue segmentation model combined with the ResNet network can realize the automatic extraction of tongue image features. The extracted features combined with machine learning modeling can be used to explore the complex hierarchical mathematical association between tongue image and clinical data. The experimental results show that the multimodal data fusion method is an important way to mine the clinical value of the TCM tongue image.

## 1. Introduction

Tongue diagnosis is an important part of Chinese medicine diagnosis, and the development of tongue diagnosis in Chinese medicine can be traced back to the Yin and Shang dynasties, after which generations of physicians have attached great importance to the application and research of tongue diagnosis, and it has been inherited as the core content of “diagnosis by looking,” which is the first of the four diagnoses in Chinese medicine. A tongue image is the observation object of tongue diagnosis, and its theoretical body is mainly derived from the theory of holistic view of Chinese medicine, which means that the physiological state of the whole body can be detected by localization [1]. Based on the holistic view of Chinese medicine, the expression of the physiological functions of the human body by the tongue can be characterized as phased, comprehensive, and dynamic. Most of the clinical studies on the Chinese medicine tongue are based on the characteristics of the tongue, such as tongue texture, tongue coating, tongue shape, and other characteristics associated with clinical diseases, which to a certain extent limits the value of the tongue to the overall expression of human physiological information. In order to realize the efficient mining of valuable vital information contained in the tongue, this study combines the current information science hotspot “deep learning” technology to explore the intelligent analysis network of tongue image and verify the practicality of the network in tongue image data mining through clinical data.

### 1.1. “End-to-End” Model of Tongue Image Data Analysis

After decades of development, the modernization of Chinese medicine tongue diagnosis has made many achievements in data acquisition and data feature extraction, but the current research difficulties are mainly focused on the discovery of clinical information of tongue images [2]. Early studies on the objectification of tongue diagnosis mostly used quantitative methods to identify tongue features and thus achieve automated classification of tongue images. In recent years, with the development of machine learning technology, the objectification of tongue diagnosis has become more clinical, and it has become possible to use tongue images to understand the diagnosis and prognosis of diseases intuitively. In 2006, Hinton and Salakhutdinov [3] proposed the concept of layered neural networks, in which there are a large number of hidden layers in these layered networks to enhance the model learning ability. It further stereotyped the neural network by using deep hidden layers to enhance the learning ability of the network for stereoscopic data such as images, speech, and video [4], allowing the network to better handle medical image data such as tongue images. Thanks to the advancement of machine learning modeling, it is possible to mine clinical data of tongue images in an “end-to-end” mode from the input of the original image captured to the output of clinical data. This changes the traditional research paradigm of associating tongue images with clinical data.

### 1.2. Network Architecture for Intelligent Analysis of Tongue Clinical Information

Intelligent analysis of tongue clinical information refers to the separation of the tongue in the original image, then feature extraction of the target region of the tongue, and modeling analysis with clinical indicators, and finally yielding a prediction model of clinical indicators based on the tongue image. In this study, based on the data characteristics of clinical test indicators, which are mainly continuous variables, an intelligent tongue analysis network is constructed using a “dual-flow” network architecture. The network is composed of four different functional module groups (Figure 1).

One is the Unet tongue segmentation network model developed by our group [5], which is a deep learning network model consisting of 11 “convolution-pooling” layers (Figure 2). The semantic segmentation test results show that the model achieves a mean intersection ratio (MIoU) of 91% and a pixel accuracy (PA) of 93%.

The second is the feature extraction module for ResNet image data. In this module, data feature vector extraction is performed by multilayer residual network (ResNet) using pretrained weight values from ImageNet dataset. The ResNet structure is designed with 8 modules, connecting a convolutional layer from the input layer in turn, and then connecting Bottleneck1-4 modules, with a 1^*∗*^1 average pooling at the end of the Bottleneck4 output connection network to retain more coding information (Figure 3).

The third is the convolutional fusion module. To meet the need for further data mining, a convolutional fusion module is set up in the network architecture to integrate the tongue image with the associated data, and the fused data can be output as independent variables for regression modeling analysis. In this module, the collected clinical data are adjusted to 1^*∗*^2048 vectors by replication expansion, and then superimposed with the 1^*∗*^2048 vectors extracted by the above ResNet network, i.e., each vector channel is D before fusion and 2D after fusion. After completing the connection fusion, a 1^*∗*^1 convolutional kernel is used to do the dimensionality reduction in the channel dimension. The data obtained by convolutional fusion for the tongue image can be combined with a certain clinical data parameter to form a multimodal fusion data structure into the end-of-network regression analysis session.

The fourth is the regression modeling analysis part at the end of the network, which uses the tongue data features or the fused data of tongue data features and a certain clinical information as independent variables to carry out the prediction of the target physiological information. The regression analysis can select multiple machine learning models according to the data type, distribution pattern, and other characteristics combined with clinical information.

## 2. Web Application Experiment of Intelligent Analysis of Tongue Image Based on Deep Learning Technology

The tongue, as a muscular organ, in a healthy state, has a light red color due to the abundance of internal capillaries, i.e., the light red tongue image. In the pathological state, on the other hand, the tongue can take on a dark or light reddish-red, purple-dark, greenish-gray, or pale white color due to factors such as the amount of hemoglobin, impaired vascular circulation, or structural problems [6]. In Su Wen - Yin Yang Ying Xiang Da Lun, “The heart is the master of the tongue …… in the orifice for the tongue”; In Ling Shu - Pulse Degree, “The heart is connected to the tongue, the heart and the tongue can know the five tastes,” on the basis of which later medical practitioners further condensed the relationship between the tongue and the heart as “the heart opens the orifice in the tongue, the tongue is the seedling of the heart.” In recent years, it has been found that the initial pathological changes of primary hypertensive disease are mostly intermittent spasms of tiny arteries throughout the body [7], which can lead to organ damage after a period of time and the initial damage sites are mainly concentrated in the tiny arteries [8]. Microvascular lesions within the tongue can have an impact on tongue color, and the tongue, as a dense area of microcirculation in the body, has a complex intertwined network of vessels at all levels [9]. It is clear that changes in arterial blood pressure in the human body first affect the microcirculatory system, and the human tongue is the largest dense organ of microcirculation that we can visually and noninvasively observe, suggesting here that there may be some correlation between tongue image and human blood pressure.

To further explore the application value of the intelligent analysis network of tongue images, a clinical experiment was set up in this study to combine the abovementioned Chinese medicine and modern medical theories for the constructed clinical data analysis network model of tongue images. The experiment was conducted with the mean value of the blood pressure values of the last 6 days of the week with staging diagnostic value as described in the Chinese Guidelines for the Prevention and Treatment of Hypertension 2018 Revision [2] as the target, and the blood pressure values of the day were collected using the tongue image and the tongue image overlay as the independent variables for the prediction experiment. To ensure the reliability and traceability of the experimental data and to reduce some interfering factors, the study population was selected from inpatients with type 2 diabetes mellitus in the Department of Endocrinology of the Affiliated Hospital of Chengdu University of Chinese Medicine. The input data of the dual-stream network were set up with two kinds of data: tongue image and blood pressure on the day of collection, and the network combined the two kinds of data into fused data by a convolutional fusion module. By comparing the prediction results of the three data, the value of tongue image in predicting the target data can be further illustrated, thus reflecting the correlation between the independent variable data and the dependent variable data to a greater extent.

The clinical trial was completed at the China Clinical Trials Registry in August 2018 (registration number: ChiCTR1800018090). The ethical review was approved by the Medical Ethics Committee of the Affiliated Hospital of Chengdu University of Traditional Chinese Medicine in July 2018 (Ethics Committee Approval Document No.: 2018KL-050). Tongue data and clinical data were collected from September 2018 to November 2019.

The tongue photo acquisition equipment used is the TFDA-1 desktop tongue diagnostic instrument developed by Shanghai University of Traditional Chinese Medicine, which consists of a CCD digital camera, LED light source, light shield, base, and curved reflector. The color temperature of the LED light is 5000K and the color rendering index is 97 as shown in Figure 4.

TFDA-1 usage and parameter settings: shooting parameters are M mode, shutter speed is 1/125; aperture value is F6.3; ISO sensitivity is 200; image size is L 5568^*∗*^3712; central focus metering; automatic white balance. The collected raw tongue data are subject to regular quality control checks.

Clinical data were obtained from the inpatient medical record system of the Affiliated Hospital of Chengdu University of Traditional Chinese Medicine. The raw data were recorded in spreadsheet form using Microsoft Office Excel software and consisted of blood pressure records twice a day, morning and evening, during the patients' hospitalization. After collection, the data were randomly divided into training set (80%) and test set (20%) by inclusion number using Excel software.

### 2.1. Experimental Environment

The hardware configuration of the experimental computer is: Intel Core I7-9700 processor, Intel Q370 motherboard, NIVDA Geforce GT1080ti graphics card; the operating system is Ubuntu 9.04, the programming language is Python 3.7, and the model network is built through pytorch.

### 2.2. Regression Analysis

Since the data consisted of three categories, the regression modeling was performed in three groups, with each group modeling diastolic blood pressure and systolic blood pressure separately. The regression models used were identical for all three data categories, and only the input independent variables were changed in the experiment. The regression analysis process of the four models is described in detail in the following section, using “blood pressure on the day” as the independent variable, which is used as a reference for the other two data categories. The sample size of the training set used in this experiment was 260 cases. Since the blood pressure data were divided into diastolic and systolic blood pressure, we modeled the prediction of diastolic blood pressure and systolic blood pressure separately, so the methods used are exactly the same, and we will not describe the methods separately, but use “blood pressure” in the following.

### 2.3. Random Forest (RF)

Random forests are reinforced classifiers consisting of multiple decision trees. The basic architecture is to form a model group of multiple decision tree classifiers and to “vote” on the output of these decision trees to determine the most optimal data processing result by the most votes [10]. A random forest of 10 trees was used for the regression experiments. The model training process is as follows:

1. The value of blood pressure on the first day of the count is taken as the independent variable, *x*_*i*_, and the mean of the patient's data from the second to the seventh day is taken as the dependent variable, *y*_*i*_.
2. For *i* = 1,2,…, 260, the training set is randomly sampled for the *i*th time and a total of 260 acquisitions are made to obtain a sample set *D*_*i*_ containing 260 blood pressure data samples, and the *i*th tree model *T*_*i*_(*x*) is trained with the sample *D*_*i*_. When training the tree model nodes, the features of some samples are randomly selected from all the blood pressure sample features on the nodes at the same time, and then an optimal feature is selected from them to be the left and right subtree division feature of the tree.
3. The abovementioned tree model is averaged out, and the arithmetic average is considered directly here, so that the final output model *L*(*x*) = 1/260∑_*k*=1_^260^*T*_*k*_(*x*) is the result.

### 2.4. Adaptive Enhancement Algorithm (AdaBoost)

The adaptive boosting algorithm (AdaBoost) is trained with multiple weak classifiers in the training set and the sample weights are corrected according to the classifier error rate and then given to the next classifier, which forms a strong classification by combining multiple sets of weak classifiers [10] as follows:

(1) Initialize the weight matrix *W* of the blood pressure data. Each of the 260 data is assigned a weight *w*_1_=1/260.
(2) Training the regression function *f*_*i*_. The process is as follows: if a blood pressure sample point is correctly predicted by the regression function *f*_*i*_, the corresponding weight is reduced for the next blood pressure training, and if it is incorrectly classified, the corresponding weight is increased. The updated blood pressure set is used to train the next classifier, and so on iteratively. In this case, the error of the regression function *f*_*i*_ is
  (1) $$\begin{array}{c} e_{t}=\sum_{i=1}^{260}w_{ii}I\left(H_{t}\left(x_{i}\right)\neq y_{i}\right), \end{array}$$
where *I*(·) is the information function, *H*(·) is the entropy function, and *W*_*ii*_ is the weight of the *i*th iteration.
(3) The obtained regression function is combined, which is the final regression function:
  (2) $$\begin{array}{c} D_{t+1}=\frac{D_{t}\left(i\right)\exp\left(-\alpha_{t}y_{i}H_{t}\left(x_{i}\right)\right)}{Z_{t}}, \end{array}$$

where $Z_{t}=2\sqrt{e_{t}\left(1-e_{t}\right)}$ is the normalization constant.

### 2.5. Iterative Decision Tree (GBRT)

GBRT is an integrated model consisting of numerous decision trees of shallow depth combined in a hierarchical connection [11], and the characteristics of GBRT are mainly focused on strong adaptability to various data categories and high accuracy of regression prediction, which is in line with the experimental design of this experiment in which prediction is carried out based on different categories of data. The decision tree model in the model group does not play the role of classification judgment, but carries out regression prediction, and this prediction process is carried out in each regression tree for the input data and more accurate prediction values are obtained through continuous correction. The calculation process in the experiment is as follows:

   Input: Blood pressure data set. *D*={(*x*_1_, *y*_1_),…, (*x*_260_, *y*_260_)}
   Output: Return to lifting tree. *T*_*D*_(*x*)
(1) Initialization *T*_0_(*x*)=0.
(2) For *n* = 1,…, 260, the residual *r*_*ni*_=*y*_*i*_ − *T*_*n*−1_(*x*_*i*_) is calculated, and the residual is fitted to obtain the regression tree as *T*(*x*; Θ_*m*_) , and the update law as *T*_*m*_=*T*_*m*−1_+*T*(*x*; Θ_*m*_).
(3) Obtaining regression tree *T*_*D*_(*x*)=∑_*m*=1_^260^*T*(*x*; Θ_*m*_).

### 2.6. Support Vector Regression (SVR)

SVR is a regression analysis, so there is only one type of sample points, and the total deviation of all sample points from the hyperplane is found to be the minimum distance in the regression process. For the consideration of linear distribution of blood pressure data, the kernel function is chosen as a linear type in this experiment. Moreover, *C* = 1*e*3, C represents the importance for outlier points. *γ*=0.01 denotes the coefficient of the kernel function, which is too large to cause overfitting because it is a linear function, and is finally chosen to be 0.01. The blood pressure data are equivalent to solving the following constrained optimization problem in the SVR:

(3) $$\begin{array}{c} \left\{\begin{array}{c} \underset{w,b}{\min}\frac{1}{2}{\left\|w\right\|}^{2},\\ \text{s.t. }\left|y_{i}-\left(wx_{i}+b\right)\right|\leq \varepsilon \;i=1,2,\ldots ,N, \end{array}\right. \end{array}$$

where **w**=*w* ∈ *R* is the weight of the regression curve and *ε* is the maximum value of the distance from the curve to the blood pressure data point.

### 2.7. Evaluation Methods of Prediction Results

There are two commonly used regression prediction evaluation methods, namely, mean absolute error (MAE) and root mean square error (RMSE). In this experiment, mean absolute error [12] (MAE) was chosen to evaluate the test results, and the mean absolute error is the absolute average of the error between the prediction results and the real data, and the larger the mean absolute error is, the worse the prediction accuracy is proved to be. The use of MAE as a criterion for judging the error can better express the true error of data with 1-dimensional characteristics compared to RMSE [13] and facilitate the comparison between different data categories. The MAE formula is as follows:

(4) $$\begin{array}{c} \text{MAE}=\frac{1}{m}\sum_{i=1}^{m}{\left\|y_{\text{test}}^{\left(i\right)}-{\hat{y}}_{\text{test}}^{\left(i\right)}\right\|}_{1}. \end{array}$$

## 3. Results

### 3.1. Data Acquisition Results

A total of 429 samples were collected according to the standardized data collection protocol described above, and 325 samples were screened after quality control to meet the study requirements, including 131 female samples and 194 male samples. The general statistics of the patients were as follows Tables 1–4.

### 3.2. Model Prediction Results

In this experiment, we used three kinds of data: “blood pressure of the day,” “blood pressure of the day + tongue,” and “tongue,” and used four kinds of end-of-data regression models to predict the 6-day average of blood pressure. The prediction accuracy was assessed by the mean absolute error. The results are shown in Tables 5 and 6.

From the prediction trend, it was found that the prediction error performance was higher for the tongue data; the prediction error results were better for the blood pressure on the day of shooting than for the tongue data. The best prediction results were obtained with the fusion data of tongue image overlaid with blood pressure on the day of shooting.

In this study, the value of tongue image in the prediction of blood pressure stage mean was evaluated using the prediction results of the same-day blood pressure data modeling as a baseline. When the mean absolute error (MAE) of the same algorithmic model from the “same-day blood pressure + tongue” and “tongue” data categories was lower than that of the “same-day blood pressure” model, it represented an improved value. On the contrary, if the MAE is higher than that of the “same-day blood pressure” model, it means that it has no value for blood pressure prediction. The prediction results showed that the MAE of each of the six predictions of systolic and diastolic blood pressure based on the “tongue image” data alone exceeded the prediction of blood pressure on the same day, and there was no significant advantage of using the tongue image alone to predict blood pressure for the next 6 days. The MAE of the model built with the fused tongue and blood pressure data was lower than that of the current day's blood pressure modelin (Figures 5 & 6).

## 4. Discussion

In this experiment, we used a dual-input “two-stream network” analysis architecture for the two types of input data to perform blood pressure stage prediction using tongue image, current day blood pressure, and both fused data. The network is designed to use the “blood pressure of the day” prediction results as the baseline, and the cross-sectional comparison of the prediction results can further reflect the contribution of different data categories in prediction accuracy. The models constructed from the fused data outperformed the models constructed from the same-day blood pressure data in all prediction results. The addition of tongue data contributes to the reduction of the error rate. Since the machine learning technique used is a “black-box” data processing model with uninterpretable complex hierarchical mathematical relationships, it is not possible to know which feature of the tongue data has a positive effect on the prediction of blood pressure. Here, this study argues that data convolution fusion makes the overall linear distribution of the fused data. The tongue image data, on the other hand, makes the amount of information increased by incorporating the information carried by features such as tongue morphology, color, and texture, which enhances the characteristics of the dimensionality of the data to some extent. Thus, the fused data incorporate a lot of lingual information compared to the same-day blood pressure data or the lingual image data only, and the overall data are still linearly distributed, which may be the reason why the fused data model is smaller than the two separate data models in terms of error. Through the above experiments, this study concluded that the multimodal data fusion method of “tongue +” mode can achieve more efficient data mining than the analysis of tongue data only. In the future, with the upgrade of data analysis capability, the tongue diagnosis data can be fused with various clinical data to form a big data matrix, and then the neural network can be used to carry out deep data mining, and its application will cover the auxiliary identification of Chinese medicine, physical determination, and the prognosis assessment of clinical indicators, radiotherapy, chemotherapy, and surgery in modern medicine.

## 5. Conclusion

Tongue diagnosis is an important part of Chinese medicine diagnosis, and the development of tongue diagnosis in Chinese medicine can be traced back to the Yin and Shang dynasties, after which generations of physicians have attached great importance to the application and research of tongue diagnosis, and it has been inherited as the core content of “diagnosis by looking,” which is the first of the four diagnoses in Chinese medicine. The experimental results show that the tongue image overlaying the current day blood pressure can improve the prediction accuracy compared with the current day blood pressure data alone, suggesting the contribution of the tongue image to the improvement of the prediction accuracy and confirming that the data fusion model is an important way to explore the clinical value of the Chinese medicine tongue image.

## Figures and Tables

**Figure 1:** Dual path network architecture diagram.

**Figure 2:** Unet tongue segmentation model.

**Figure 3:** ResNet network structure.

**Figure 4:** TFDA-1 benchtop tongue diagnostic instrument.

**Figure 5:** Comparison of mean absolute error in predicting systolic blood pressure prediction.

**Figure 6:** Comparison of mean absolute errors in predicted diastolic blood pressure.

**Table 1:** Age distribution of subjects.

*N*	Age	Max.	Min.

325	49.04 ± 13.50	75	34

**Table 2:** Distribution of subject's height (cm).

Gender (*N*)	Height	Max.	Min.

Male (194)	169.48 ± 5.76	185	153
Female (131)	157.12 ± 5.76	173	145

**Table 3:** Distribution of subjects' weight (kg).

Gender (*N*)	Weight	Max.	Min.

Male (984)	68.76 ± 16.72	120	49
Female (1064)	157.71 ± 5.97	95	41

**Table 4:** Subjects' education status.

Education level	*N*	Percentage

University	45	13.84%
High school (secondary school)	153	47.08%
Other	127	39.08%

**Table 5:** Mean absolute error of predicted systolic blood pressure (MAE) in mmHg.

Model data	SVR	RF	Adaboost	GBRT

Blood pressure for the day	7.13	6.54	5.91	6.25
Tongue image	15.41	10.39	10.22	9.61
Tongue image + blood pressure on the day	7.06	**5.49**	5.54	5.84

**Table 6:** Mean absolute error of predicted diastolic blood pressure (MAE) in mmHg.

Model Data	SVR	RF	Adaboost	GBRT

Blood pressure for the day	7.10	8.61	4.43	6.17
Tongue image	18.03	13.91	11.87	15.73
Tongue image + blood pressure on the day	6.32	8.54	**4.02**	5.91

## Data Availability

The numerical dataset used to perform the study presented in the paper are available from the corresponding author upon request.
